The article "Inflammation and Oxidative Stress Role of S100A12 as a Potential Diagnostic and Therapeutic Biomarker in Acute Myocardial Infarction" was retracted in 2023. Reasons: signs of a paper mill; compromised peer review; unreliable results or conclusions.

# Inflammation and Oxidative Stress Role of S100A12 as a Potential Diagnostic and Therapeutic Biomarker in Acute Myocardial Infarction

**DOI:** 10.1155/2022/2633123

**Published:** 2022-08-25

**Authors:** Jian Xie, Changjun Luo, Binhai Mo, Yunhua Lin, Guoqing Liu, Xiantao Wang, Lang Li

**Affiliations:** ^1^Department of Cardiology, The First Affiliated Hospital of Guangxi Medical University, Guangxi Cardiovascular Institute, Nanning, 530021 Guangxi, China; ^2^Department of Cardiology, The First People Hospital of Nanning & The Fifth Affiliated Hospital of Guangxi Medical University, Nanning, 530016 Guangxi, China; ^3^The First Clinical Medical College, Guangxi Medical University, Nanning 530021, China; ^4^Guangxi Key Laboratory of Precision Medicine in Cardio-Cerebrovascular Diseases Control and Prevention, Nanning, 530021 Guangxi, China

## Abstract

Acute myocardial infarction (AMI) is one of the most serious cardiovascular diseases with high morbidity and mortality. Numerous studies have indicated that S100A12 may has an essential role in the occurrence and development of AMI, and in-depth studies are currently lacking. The purpose of this study is to investigate the effect of S100A12 on inflammation and oxidative stress and to determine its clinical applicability in AMI. Here, AMI datasets used to explore the expression pattern of S100A12 in AMI were derived from the Gene Expression Omnibus (GEO) database. The pooled standard average deviation (SMD) was calculated to further determine S100A12 expression. The overlapping differentially expressed genes (DEGs) contained in all included datasets were recognized by the GEO2R tool. Then, functional enrichment analyses, including Gene Ontology (GO) and Kyoto Encyclopedia of Genes and Genomes (KEGG) analyses, were carried out to determine the molecular function of overlapping DEGs. Gene set enrichment analysis (GSEA) was conducted to determine unrevealed mechanisms of S100A12. Summary receiver operating characteristic (SROC) curve analysis and receiver operating characteristic (ROC) curve analysis were carried out to identify the diagnostic capabilities of S100A12. Moreover, we screened miRNAs targeting S100A12 using three online databases (miRWalk, TargetScan, and miRDB). In addition, by comprehensively using enzyme-linked immunosorbent assay (ELISA), real-time quantitative PCR (RT–qPCR), Western blotting (WB) methods, etc., we used the AC16 cells to validate the expression and underlying mechanism of S100A12. In our study, five datasets related to AMI, GSE24519, GSE60993, GSE66360, GSE97320, and GSE48060 were included; 412 overlapping DEGs were identified. Protein-protein interaction (PPI) network and functional analyses showed that S100A12 was a pivotal gene related to inflammation and oxidative stress. Then, S100A12 overexpression was identified based on the included datasets. The pooled standard average deviation (SMD) also showed that S100A12 was upregulated in AMI (SMD = 1.36, 95% CI: 0.70-2.03, *p* = 0.024). The SROC curve analysis result suggested that S100A12 had remarkable diagnostic ability in AMI (AUC = 0.90, 95% CI: 0.87-0.92). And nine miRNAs targeting S100A12 were also identified. Additionally, the overexpression of S100A12 was further confirmed that it maybe promote inflammation and oxidative stress in AMI through comprehensive in vitro experiments. In summary, our study suggests that overexpressed S100A12 may be a latent diagnostic biomarker and therapeutic target of AMI that induces excessive inflammation and oxidative stress. Nine miRNAs targeting S100A12 may play a crucial role in AMI, but further studies are still needed. Our work provides a positive inspiration for the in-depth study of S100A12 in AMI.

The article "Inflammation and Oxidative Stress Role of S100A12 as a Potential Diagnostic and Therapeutic Biomarker in Acute Myocardial Infarction" was retracted in 2023. Reasons: signs of a paper mill; compromised peer review; unreliable results or conclusions.

## 1. Introduction

As a serious heart disease, acute myocardial infarction (AMI) has the characteristics of high mortality and a poor prognosis; and it is easy to induce severe cardiovascular events, such as ventricular remodeling and heart failure, which seriously threaten people's lives and cause great pain and financial burden in patients [1–3]. The early diagnosis and treatment of AMI are essential for reducing myocardial injury and malignant consequences, reducing mortality and improving patient prognosis to some extents [4–6]. Currently, the levels of myocardial enzyme (CKMB) and cardiac troponin I (cTnI) are still the gold standards for the clinical diagnosis of AMI, but they are not specific for AMI. Previous studies indicated that patients with heart failure, chronic kidney disease, and septicemia also have elevated cardiac troponin I (cTnI) levels, which may lead to false-positive results in AMI diagnosis [7, 8]. Current studies have suggested that the circulating miRNAs, such as miRNA-499, miRNA-22, miR-223-3p, and miR-483-5p, could be used as potential biomarkers of AMI [9–11]. However, there are still few biomarkers available in the clinic; thus, identifying new biomarkers that can be used in the diagnosis and treatment of AMI is still imperative.

AMI can lead to cardiomyocyte death, often followed by a robust inflammatory response in myocardial tissue. Previous studies have demonstrated that the activation of complement and Toll-like receptor (TLR)/interleukin-1 (IL-1) signaling is involved in the onset and development of inflammation [12–14]. A suitable inflammatory response is beneficial for the healing of injured myocardial tissue, indicating that the body performs the function of self-repair. However, a persistent excessive inflammatory response further aggravates cardiomyocyte apoptosis and may lead to serious adverse events, such as arrhythmia, which seriously affect patient prognosis [15, 16]. In addition, the pathogenesis of AMI is associated with the excessive production of reactive oxygen species (ROS), which induce oxidative stress. Oxidative stress is the main cause of the poor prognosis of ischemic myocardial injury in AMI [17]. Several other studies have also identified oxidative stress as a key factor in AMI [18–20]. Therefore, therapy that targets inflammation and oxidative stress may become a potential treatment strategy for patients with AMI.

The article "Inflammation and Oxidative Stress Role of S100A12 as a Potential Diagnostic and Therapeutic Biomarker in Acute Myocardial Infarction" was retracted in 2023. Reasons: signs of a paper mill; compromised peer review; unreliable results or conclusions.

S100 calcium-binding protein A12 (S100A12) is a calcium-binding protein that plays a vital role in various diseases [21]. In ischemia-reperfusion (I/R) injury, S100A12 promotes inflammation, oxidative stress, and apoptosis by activating ERK signaling in vitro [22]. In addition, S100A12 was identified to be involved in the development of atherosclerosis through the S100A12-CD36 axis, and its expression was upregulated in unstable plaques [23]. It was also previously reported that tumor necrosis factor alpha (TNF-*α*)+S100A12 treatment stimulated nicotinamide adenine dinucleotide phosphate (NADPH) oxidase activity and the production of hydrogen peroxide (H2O2) in human aortic smooth muscle cells (HASMCs) [24]. The above evidence suggests that S100A12 plays an essential part in inflammation and oxidative stress in numerous diseases. However, few existing reports concern the expression, potential mechanism, and clinical significance of S100A12 in AMI. Tong et al. identified 10 gene signatures, including S100A12, as effective markers for diagnosing AMI [25]. Zhang et al. reported S100A12 was a novel diagnostic biomarker for the identification of patients with ST-elevation myocardial infarction (STEMI) [26]. In addition, Gobbi et al. constructed a logical regression model containing five platelet gene expression datasets (FKBP5, S100P, SAMSN1, CLEC4E, and S100A12) that can identify STEMI and healthy donors [27]. But the above studies did not elucidate the underlying mechanism of S100A12 in AMI, especially those related to inflammation and oxidative stress, and the reliability of some studies was limited by insufficient sample sizes. Therefore, our study is the first to integrate public data and in vitro experiments to comprehensively explore its potential mechanism in inflammation and oxidative stress and its clinical application value in AMI.

In our current study, the expression pattern, potential mechanism, and clinical significance of S100A12 in AMI were probed using public datasets. Based on bioinformatics methods, potential miRNAs targeting S100A12 were predicted via three online databases (miRWalk, TargetScan, and miRDB). Furthermore, a series of in vitro experiments were carried out to elucidate the effect of S100A12 on inflammation and oxidative stress in AMI. In summary, this study reveals that overexpressed S100A12 is involved in inducing excessive inflammation and oxidative stress and could be applied as a feasible diagnostic biomarker and prospective therapeutic target related to inflammation and oxidative stress in AMI.

The article "Inflammation and Oxidative Stress Role of S100A12 as a Potential Diagnostic and Therapeutic Biomarker in Acute Myocardial Infarction" was retracted in 2023. Reasons: signs of a paper mill; compromised peer review; unreliable results or conclusions.

## 2. Materials and Methods

### 2.1. Overall Study Design and Flow

Here, we first explored the expression pattern and clinical significance of S100A12 in AMI using public data and conducted Gene Ontology (GO) analysis, Kyoto Encyclopedia of Genes and Genomes (KEGG) analysis, and Gene set enrichment analysis (GSEA) to explore its possible mechanism. Furthermore, real-time quantitative PCR (RT–qPCR), enzyme-linked immunosorbent assay (ELISA), Western blotting (WB) methods, and other in vitro experiments were carried out to verify the effect of S100A12 in AMI. The overall design and flow diagram of this study are presented in Figure 1.

### 2.2. GEO Dataset Downloading and Data Preprocessing

All AMI expression profile datasets were obtained through the Gene Expression Omnibus (GEO) database (https://www.ncbi.nlm.nih.gov/geo/). We searched for the gene expression profile data of AMI in the GEO database and screened the identified datasets according to the inclusion and exclusion criteria. The inclusion criteria were as follows: (1) including three or more pairs of samples from an AMI group and a non-AMI group and (2) derived from a human source. The exclusion criteria were as follows: (1) that data could not be downloaded and (2) no complete gene expression profile data were provided. Finally, five datasets (GSE24519, GSE60993, GSE66360, GSE97320, and GSE48060) that were included in the standard and did not meet the exclusion criteria were included in this study. The dataset information was described in detail in Table 1. Furthermore, all data downloaded from the GEO database were transformed into log2 values for further analysis. And we integrated all included datasets using the “sva” R package and removed batch effects to form a merged dataset.

### 2.3. Screening of Overlapping Differentially Expressed Genes (DEGs) via GEO2R

GEO2R, a web page interaction tool provided by the GEO database, was applied to analyze the differential expression level of genes between the AMI group and non-AMI group. In this study, four datasets, GSE24519, GSE60993, GSE66360, and GSE97320, were used as the discovery datasets to screen the overlapping DEGs using the online web tool GEO2R. Only those genes with *p* < 0.05 and log2FC < 0 were defined as downregulated DEGs. In contrast, those genes with *p* < 0.05 and log2FC > 0 were defined as upregulated DEGs. Then, the DEGs in each dataset were intersected and defined the overlapping genes as the final overlapping DEGs. Notably, the GSE48060 dataset contained information regarding the recurrence condition of AMI patients; thus, this dataset was not included in the discovery dataset, which was used to evaluate the ability of S100A12 to distinguish between recurrent and nonrecurrent patients.

The article "Inflammation and Oxidative Stress Role of S100A12 as a Potential Diagnostic and Therapeutic Biomarker in Acute Myocardial Infarction" was retracted in 2023. Reasons: signs of a paper mill; compromised peer review; unreliable results or conclusions.

### 2.4. Functional Analysis of Overlapping DEGs and S100A12

KEGG and GO analyses were carried out through the Database for Annotation, Visualization, and Integrated Discovery (DAVID) (version 6.8, https://david.ncifcrf.gov/) to comprehensively understand the potential biological functions and pathways of the overlapping DEGs. To visualize the analysis results, the enrichment results of the top 12 genes (based on the number of enrichment genes) in the KEGG and GO enrichment analyses were intuitively presented as bar charts. Furthermore, the merged dataset was divided into high and low expression groups based on the median expression value of S100A12, and then, a GSEA analysis was carried out using GSEA software (version 4.1.0) to clarify its potential mechanism in AMI (an FDR < 0.25 and nominal *p* < 0.05 were used as the screening criteria for enriched pathways, and “c5.go.bp.v7.5.symbols.gmt” was chosen as the reference gene set used for this analysis).

### 2.5. PPI Network Analysis and Identification of Hub Genes

Protein-protein interaction (PPI) analysis is usually performed using the online tool STRING (release 11.0, http://www.string-db.org/). Based on STRING, we analyzed the PPIs of the selected overlapping DEGs and constructed a PPI network using Cytoscape 3.6.1 software. Using the cytoHubba plug-in, the overlapping DEGs with a degree of not less than 12 and ranking in the top 40 were identified as hub genes.

### 2.6. Identification of S100A12 Expression Levels in Five Datasets

By mining the online database, we obtained five datasets that provided the S100A12 gene expression profile data of AMI patients and non-AMI patients. To determine the expression pattern of S100A12 in AMI, we first explored the expression levels of S100A12 in each separate dataset, and the results were shown in the form of a scatter plot. Then, we integrated all included dataset expression profile data to comprehensively evaluate the expression levels of S100A12. As the included data were continuous variables, Stata 14 software was applied to calculate the pooled standard mean deviation (SMD). Egger's test was applied to estimate the publication bias, and *p* > 0.05 indicated no publication bias. The *Q* test and *I*^2^ statistics were used to evaluate the heterogeneity of the analysis using the random effect model under the premise of *I*^2^ > 50%. Otherwise, the fixed effect model was applied for nonsignificant heterogeneity.

The article "Inflammation and Oxidative Stress Role of S100A12 as a Potential Diagnostic and Therapeutic Biomarker in Acute Myocardial Infarction" was retracted in 2023. Reasons: signs of a paper mill; compromised peer review; unreliable results or conclusions.

### 2.7. Clinical Significance of S100A12 in AMI

To test the diagnostic ability of S100A12 in AMI, receiver operator characteristic (ROC) curves were constructed by GraphPad Prism 8 software, and the area under the curve (AUC) was calculated to assess the diagnostic ability of S100A12. Moreover, using Stata 14 software, we plotted a summary receiver operating characteristic (SROC) curve and then calculated the AUC to further identify the diagnosibility of S100A12 in AMI.

### 2.8. Prediction of miRNAs Targeting S100A12 via Multiple Databases

We used miRWalk3.0 (http://mirwalk.umm.uni-heidelberg.de/), miRDB (http://mirdb.org/), and TargetScan7.0 (http://www.targetscan.org) for the prediction of miRNAs targeting S100A12 and then obtained the chiasm of the three database predictions. Finally, S100A12 was defined as the target gene of overlapping miRNAs.

### 2.9. Verification of the Role of S100A12 Expression through In Vitro Experiments

#### 2.9.1. Model Establishment

We constructed an oxygen-glucose deprivation (OGD) model using the AC16 cells (purchased from Tongpai, Shanghai, China) as previously reported to mimic the state of cardiomyocytes in AMI in vitro [28]. Briefly, AC16 cells were initially cultured in Dulbecco's modified Eagle's medium (DMEM) (Gibco, Grand Island, NY, USA) for 24 h in a 37°C and 20% O_2_ incubator. Then, the cells were washed 3 times with phosphate-buffered saline (PBS) and incubated with glucose- and serum-free DMEM for 6 h at 37°C and 2% O_2_ to induce AMI in vitro.

#### 2.9.2. Knockdown and Overexpression of S100A12

AC16 cells were transfected with small interfering RNAs (siRNAs) specific for S100A12 and nontargeting siRNAs (Shenggong, Shanghai, China) as a negative control (Si-NC) using Lipofectamine 3000 reagent (Invitrogen, Carlsbad, CA, USA). The transfection time was 48 hours, and the concentration of siRNAs used was 50 nM [29]. In addition, S100A12 overexpression and negative control overexpression (OE-NC) plasmids (3 *μ*g) were transfected into AC16 cells. Supplementary table 1 presented the sequences of small interfering RNAs (siRNAs) and overexpression plasmids. The above experiments were carried out following the instructions supplied by the manufacturer.

The article "Inflammation and Oxidative Stress Role of S100A12 as a Potential Diagnostic and Therapeutic Biomarker in Acute Myocardial Infarction" was retracted in 2023. Reasons: signs of a paper mill; compromised peer review; unreliable results or conclusions.

#### 2.9.3. Cell Counting Kit-8 (CCK-8) Assay

CCK-8 assay was applied to determine the cell viability following the instructions provided by the manufacturer of the CCK-8 kit (Dojindo, Japan). And a microplate reader was used to read the optical density (OD) value at 490 nm.

#### 2.9.4. Quantitative Real-Time Polymerase Chain Reaction (qRT-PCR)

Total RNA was extracted from AC16 cells using TRIzol reagent (Invitrogen) based on the manufacturer's instructions. Then, the mRNA expression of S100A12 in different groups of AC16 cells was detected by RT-qPCR using the TB Green® Premix Ex Taq™ II (TaKaRa, Japan). The primer sequences used in our study were listed as follows: S100A12: upstream: 5′-TCCACCAATACTCAGTTCGGAAG-3′, downstream: 5′-ACTCTTTGTGGGTGTGGTAATGG-3′, and GAPDH: upstream: 5′-GGAGTCCACTGGCGTCTTCA-3′, downstream: 5′-GTCATGAGTCCTTCCACGATACC-3′.

#### 2.9.5. Western Blotting (WB) Analysis

To determine the protein expression level of S100A12, we used sodium dodecyl sulfate-polyacrylamide gel electrophoresis (SDS-PAGE) at a constant voltage of 100 V to separate the total protein of each group of AC16 cells, which was then transferred to polyvinylidene fluoride membranes (PVDF, Millipore, Atlanta, Georgia, United States). Subsequently, the membranes were blocked with bovine serum albumin (BSA) for 1 hour at 25°C, followed by incubation with the corresponding primary antibody (anti-S100A12, 1 : 1000, Abcam) overnight at 4°C. After 24 h, the membrane was washed five times and incubated with an enzyme-conjugated secondary antibody (1 : 1000, Abcam) for 2 h. GAPDH was used as a normalized control.

#### 2.9.6. Inflammatory Indicator Assessment

The ELISA was used to detect the expression levels of inflammation-related genes, including interleukin 1*β* (IL1-*β*) and tumor necrosis factor alpha (TNF-*α*), in each group of samples.

#### 2.9.7. Oxidative Stress Indicator Assessment

The malondialdehyde (MDA) expression levels in each group of samples were detected using an MDA assay kit (A003-1-2; Nanjing Jiancheng Bioengineering Institute, Nanjing, China) according to the manufacturer's instructions; and the intracellular reactive oxygen species (ROS) levels were determined with dichlorodihydrofluorescein diacetate (DCFH-DA) (Sigma, USA). Specifically, 50 *μ*M DCFH-DA was applied to incubate the samples for 30 min at 37°C in the dark. Then, the samples were washed twice with cold phosphate buffer (Servicebio, Wuhan, China). Immediately thereafter, a fluorescence microscope (Olympus IX51, Japan) was conducted to capture intracellular ROS fluorescence images.

### 2.10. Statistical Analysis

The comparisons between two and multiple groups were carried out using an independent samples *t*-test and a one-way analysis of variance (ANOVA), respectively. Unless otherwise specified, the number of samples per group was equal to 3 (*n* = 3). The ROC curves and scatter plots were drawn with GraphPad Prism 8 software. The SROC curve and Egger's test were performed by Stata 14 software. In R software (version 3.6.3), the visualization of the functional enrichment analyses results was performed with the application of the R package ggplot2.

The article "Inflammation and Oxidative Stress Role of S100A12 as a Potential Diagnostic and Therapeutic Biomarker in Acute Myocardial Infarction" was retracted in 2023. Reasons: signs of a paper mill; compromised peer review; unreliable results or conclusions.

## 3. Results

### 3.1. Screening of Overlapping Differentially Expressed Genes (DEGs) via GEO2R

The differential expression levels of genes in the included datasets were analyzed through the online web tool GEO2R, and the overlapping DEGs screened from 4 separate datasets (GSE24519, GSE60993, GSE66360, and GSE97320) were intersected. Ultimately, we screened a total of 412 overlapping DEGs, all of which were used for further analysis (Figure 2).

### 3.2. Functional Analysis of Overlapping DEGs and S100A12

To reveal the possible biological function and enrichment pathways of the overlapping DEGs, the KEGG pathway analysis and GO analysis were carried out. Among them, GO analysis consisted of three categories: biological process (BP), cellular component (CC), and molecular function (MF). In the BP category, the overlapping DEGs were mainly enriched in signal transduction, positive regulation of I-kappaB kinase/NF-kappaB signaling, inflammatory response, etc. (Figure 3(a)). For the CC category, the overlapping DEGs were enriched in many aspects, such as cytoplasm, cytosol, and nucleus (Figure 3(b)). For the MF category, the overlapping DEGs were significantly enriched in protein binding, ATP binding, and protein homodimerization activity (Figure 3(c)). In addition, these genes were particularly associated with butirosin and neomycin biosynthesis, the phagosome, the NF-kappaB signaling pathway, and the biosynthesis of antibiotics in the KEGG enrichment analysis (Figure 3(d)). Notably, S100A12 was the only overlapping DEGs enriched in all three aspects that were closely associated with the onset and development of inflammation, including GO:0043406~positive regulation of MAP kinase activity, GO:0006954~inflammatory response, and GO:0043123~positive regulation of I-kappaB kinase/NF-kappaB signaling (Table 2). Furthermore, the GSEA analysis showed that multiple oxidative stress-related pathways, including the regulation of the oxidative stress response, the response to oxidative stress, and regulation of oxidative stress-induced cell death, were significantly activated in the samples with high S100A12 expression (Figure 3(e)).

### 3.3. PPI Network Analysis and Identification of Hub Genes

We obtained 40 hub genes (contained S100A12; rank = 33, score = 13) according to the criteria that the degree was not less than 12 and ranked in the top 40 (Figure 4(a)). Our above study results showed that S100A12 was enriched in several classical pathways associated with inflammation and oxidative stress. Consequently, we conjectured that high expression of S100A12 may play an essential role in the occurrence and development of AMI and promote myocardial inflammation and oxidative stress, which deserves further experimental verification.

The article "Inflammation and Oxidative Stress Role of S100A12 as a Potential Diagnostic and Therapeutic Biomarker in Acute Myocardial Infarction" was retracted in 2023. Reasons: signs of a paper mill; compromised peer review; unreliable results or conclusions.

### 3.4. The Expression Levels of S100A12 in AMI

Based on the GEO database, we screened five datasets, including GSE24519, GSE60993, GSE66360, GSE97320, and GSE48060, and then, we extracted the expression level of S100A12 from five above separate datasets, and the outcomes are shown in Table 3. In addition, we intuitively showed the expression level of S100A12 in five datasets between AMI group and non-AMI group in the form of a scatter plot (Figures 4(b)–4(f)). Because of the large heterogeneity (*I*^2^ = 64.4%, *p* = 0.024; Figure 5(a)), the random effect model was carried out to calculate the SMD. The pooled SMD of S100A12 was 1.36 (95% CI: 0.70-2.03, *p* = 0.024; Figure 5(a)), indicating that the expression of S100A12 was significantly upregulated in the AMI group compared with that in the non-AMI group. Egger's test showed that there was no obvious publication bias of overexpressed S100A12 in AMI (*p* = 0.448, Figure 5(b)). In summary, all the results we obtained thus far confirmed that S100A12 was overexpressed in AMI.

### 3.5. Clinical Significance of S100A12 in AMI

We used GraphPad Prism 8 and Stata 14 software to draw ROC curves and SROC curves, respectively. An AUC value of 0.5 to 0.7 indicates a poor diagnostic value, whereas an AUC value of 0.7 to 0.9 indicates a moderate diagnostic value. A value above 0.9 suggests that the identified biomarkers have good diagnostic value [30]. The ROC results showed that the AUC values were greater than 0.7 in the five separate datasets included in this study, proving that S100A12 has upper-middle diagnostic ability (Figures 6(a)–6(e)). The SROC results indicated that S100A12 had excellent diagnosibility (AUC = 0.90, 95% CI: 0.87-0.92; Figure 5(c)). However, our results showed that S100A12 cannot effectively distinguish recurrent patients from nonrecurrent patients (AUC = 0.59, *p* = 0.52; Figure 6(f)). Nevertheless, our findings suggested that S100A12 could be used to distinguish the AMI group samples from the non-AMI group samples. S100A12 may be a diagnostic marker of AMI and has certain clinical application value.

### 3.6. Prediction of miRNAs Targeting S100A12 via Multiple Databases

After taking the intersection of the prediction results of the three databases (miRWalk, miRDB, and TargetScan), 9 miRNAs were identified, including hsamiR-4710, hsa-miR-7855-5p, hsa-miR-5589-5p, hsa-miR-4505, hsa-miR-5004-5p, hsa-miR-6858-5p, hsa-miR-1224-5p, hsa-miR-3667-5p, and hsa-miR-5787 (Figure 6(g)).

The article "Inflammation and Oxidative Stress Role of S100A12 as a Potential Diagnostic and Therapeutic Biomarker in Acute Myocardial Infarction" was retracted in 2023. Reasons: signs of a paper mill; compromised peer review; unreliable results or conclusions.

### 3.7. Validation of S100A12 Overexpression In Vitro

We successfully constructed an OGD model according to the methods described above, and the CCK-8 detection results showed that the cell viability of the OGD group was significantly lower than that of the Con (control) group (Figure 7(a)). The measurement results of the WB and qRT-PCR analyses suggested that both the protein and mRNA expression levels of S100A12 in the OGD group were significantly higher than that in the Con group (Figures 7(b)–7(d)).

### 3.8. Achieving Knockdown and Overexpression of S100A12

Both the PCR and WB results indicated that the expression of S100A12 in the Con+Si-S100A12 group was lower than that in the Con+Si-NC group (Figures 7(e)–7(g)). In contrast, its expression in the Con+OE-S100A12 group was higher than that in the Con+NC group (Figures 7(h)–7(j)). Overall, the consistent results of the PCR and WB analyses indicate that we successfully achieved knockdown and overexpression of S100A12.

### 3.9. Assessment of the Role of S100A12 Knockdown on Inflammation and Oxidative Stress in the OGD Model

The results of the CCK-8 assay (Figure 8(a)) suggest that the cell viability of the OGD+Si-S100A12 group was higher compared with the OGD+Si-NC group (*p* < 0.05). In addition, the expression levels of S100A12 (Figures 8(b) and 8(c)), inflammatory indicators (TNF-*α* and IL1-*β*) (Figures 8(d) and 8(e)), and oxidative stress indicators (ROS and MDA) in the OGD+Si-NC group were significantly increased compared with the OGD+Si-S100A12 group (*p* < 0.05) (Figure 8(f)–8(g)). Therefore, we concluded that the knockdown of S100A12 expression could alleviate inflammation and oxidative stress in the OGD model and reduce cardiomyocyte injury.

### 3.10. Assessment of the Role of S100A12 Overexpression on Inflammation and Oxidative Stress in the OGD Model

The results of the CCK-8 assay (Figure 9(a)) suggest that the cell viability of the OGD+OE-S100A12 group samples was lower compared with the OGD+NC group (*p* < 0.05). In addition, the expression levels of S100A12 (Figure 9(b) and 9(c)), inflammatory indicators (TNF-*α* and IL1-*β*) (Figures 9(d) and 9(e)), and oxidative stress indicators (ROS and MDA) in the OGD+OE-S100A12 group were significantly increased compared with the OGD+NC group (*p* < 0.05) (Figures 9(f) and 9(g)). The above evidence concluded that S100A12 overexpression aggravated inflammation and oxidative stress in the OGD model, leading to cardiomyocyte injury.

The article "Inflammation and Oxidative Stress Role of S100A12 as a Potential Diagnostic and Therapeutic Biomarker in Acute Myocardial Infarction" was retracted in 2023. Reasons: signs of a paper mill; compromised peer review; unreliable results or conclusions.

## 4. Discussion

Acute myocardial infarction (AMI) is one of the most serious cardiovascular diseases, an early diagnosis of AMI is very important, but diagnostic biomarkers and therapeutic targets available in the clinic are lacking [31–33]. Inflammation and oxidative stress are involved in adverse outcomes of AMI [34–37]. As a member of the S100 protein family, S100A12 has been confirmed to play a role in various cardiovascular disease [38–42]. However, there are still few studies systematically exploring the role and potential application value of S100A12 in AMI through integrated means of bioinformatics and experimental validation, especially its effects on inflammation and oxidative stress. Therefore, we attempted to identify a potential diagnostic biomarker and therapeutic target associated with inflammation and oxidative stress through bioinformatics techniques and multiple in vitro experiments.

Our study suggested that the mitogen-activated protein kinase (MAPK) signaling pathway, NF-kappaB signaling pathway, and inflammatory response pathway, which S100A12 was enriched in, were associated with the occurrence and development of AMI. MAPK can be divided into four subfamilies, extracellular signal-regulated kinase (ERK), p38, c-Jun N-terminal kinase (JNK), and ERK54 that participate in many biological processes, such as cell proliferation, apoptosis, and inflammation [43]. The p38 MAPK signaling pathway played a vital role in the secretion and activity of TNF-*α*, IL-2, IL-1, and other proinflammatory cytokines in human endothelial cells. ERK1/2 phosphorylation mediates myocardial fibrosis induced by transforming growth factor-*β*1 by activating Rho kinase1 in myocardial infarction model rats [44]. The JNK-NF-kappaB signal transduction cascade could be inhibited by the intrinsic activation of AMP-activated protein kinase (AMPK), thereby reducing ischemia/reperfusion-induced inflammation [45]. The NF-kappaB signaling pathway was closely related to the occurrence of inflammation. A study reported that adiponectin inhibited the activation of the NF-kappaB signaling pathway and the expression of proinflammatory genes, thereby inhibiting the inflammatory response in atherosclerosis [46]. Moreover, Zhang et al. confirmed that S100A12 could promote inflammation induced by ischemia-reperfusion injury by activating ERK signal transduction [22]. The GSEA analysis further suggested that overexpressed S100A12 may be associated with excessive oxidative stress. Previous studies have suggested that the oxidative stress levels are significantly elevated in AMI, which could cause myocardial cell dysfunction and damage [47, 48]. In addition, excessive oxidative stress and an inflammatory response could promote the occurrence of heart failure in patients with AMI [49]. Based on the above evidence, we speculated that S100A12 may promote the inflammatory response, oxidative stress, and myocardial damage after AMI.

The article "Inflammation and Oxidative Stress Role of S100A12 as a Potential Diagnostic and Therapeutic Biomarker in Acute Myocardial Infarction" was retracted in 2023. Reasons: signs of a paper mill; compromised peer review; unreliable results or conclusions.

Furthermore, nine miRNAs targeting S100A12, including hsamiR-4710, hsa-miR-7855-5p, hsa-miR-5589-5p, hsa-miR-4505, hsa-miR-5004-5p, hsa-miR-6858-5p, hsa-miR-1224-5p, hsa-miR-3667-5p, and hsa-miR-5787, were predicted via three online databases (miRWalk, TargetScan, and miRDB). hsa-miR-5787 inhibited inflammation mediated by macrophages in ischemic cerebral infarction through regulating TLR4/NF-kappaB signaling [50]. hsa-miR-4505 aggravated lipopolysaccharide- (LPS-) induced vascular endothelial cell injury by regulating heat shock proteinA12B (HSPA12B) [51]. Moreover, it was reported that hsa-miR-1224-5p, hsa-miR-4710, and hsa-miR-7855-5p played important roles in various cancers. For example, hsa-miR-1224-5p inhibited the proliferation and invasion of ovarian cancer by targeting staphylococcal nuclease and tudor domain containing 1 (SND1) [52]; hsa-miR-4710 could be used to predict axillary lymph node metastasis of breast cancer [53]. The expression of hsa-miR-7855-5p could be downregulated due to the overexpression of AC006262.5, which ultimately promoted the proliferation and migration of hepatocellular carcinoma [54]. However, few studies focused on hsa-miR-6858-5p, hsa-miR-5004-5p, hsa-miR-3667-5p, and hsa-miR-5589-5p, especially in cardiovascular diseases. Generally, the molecular mechanism of these nine miRNAs and their relationship with S100A12 in AMI are still unclear and need to be further studied.

Moreover, we comprehensively used public data and in vitro experiments of S100A12 expression, its clinical significance, and its effect on inflammation and oxidative stress in AMI. The research based on public data preliminarily showed that S100A12 expression was upregulated in AMI and has a good diagnostic value for AMI. The in vitro experiments confirmed that the expression of S100A12 was significantly upregulated in AMI (OGD model), and its overexpression promoted the occurrence of inflammation and oxidative stress, while the knockdown of its expression had the opposite effect. Several studies have also shown that inhibiting inflammation and oxidative stress can alleviate myocardial damage caused by myocardial infarction. Zhang et al. demonstrated that the inhibition of death-associated protein kinase 1 (DAPK1) expression inhibited inflammation and oxidative stress and protected rats from myocardial injury caused by myocardial infarction [55]. In addition, a study by Xiao et al. showed that the overexpression of lung cancer associated transcript 1 (LUCAT1) has a protective effect on AMI by inhibiting the effects of H_2_O_2_ on oxidative stress, inflammation, viability, and apoptosis in H9c2 cells [56]. Therefore, we speculate that inhibiting the expression of S100A12 could inhibit oxidative stress and inflammation, thereby exerting a similar cardioprotective effect and reducing myocardial injury. S100A12 is expected to serve as a novel target for the diagnosis and treatment of AMI injury, providing clinical benefits to patients.

The article "Inflammation and Oxidative Stress Role of S100A12 as a Potential Diagnostic and Therapeutic Biomarker in Acute Myocardial Infarction" was retracted in 2023. Reasons: signs of a paper mill; compromised peer review; unreliable results or conclusions.

However, there are some limitations in this study that affect the dependability of our research results. Initially, the AMI dataset was not as easy to obtain as a tumor dataset, and there are few AMI expression profile datasets in the GEO database, leading to a small research sample size and reducing the accuracy of our research. Second, the large sample size difference in some datasets affects the accuracy of our statistical analysis to a certain extent. Third, more deeper in vivo and vitro experiments should be carried out to carefully verify our results. Although we conducted in vitro experiments to demonstrate that S100A12 overexpression promotes inflammation and oxidative stress, future in vitro and in vivo experiments with larger sample sizes are still needed to explore the specific molecular mechanisms.

## 5. Conclusion

In summary, our study revealed high expression of S100A12 in AMI and its positive regulation of inflammation and oxidative stress using bioinformatics methods and comprehensive analysis of in vitro experiments. S100A12 may contribute to the early diagnosis of AMI, and inhibiting its expression may reduce myocardial damage and benefit the treatment of AMI patients. And we also identified 9 miRNAs targeting S100A12. Our study can provide certain reference value for further research on the role of S100A12 in the diagnosis and treatment of AMI.

## Figures and Tables

**Figure 1:** Overall design and flow chart of this study. Notes: AMI: acute myocardial infarction; S100A12: S100 calcium-binding protein A12; KEGG: Kyoto Encyclopedia of Genes and Genomes; GO: Gene Ontology; SMD: standardized mean difference; ROC: receiver operating characteristic; SROC: summary receiver operating characteristic; GSEA: gene set enrichment analysis; RT-qPCR: real-time quantitative PCR; ELISA: enzyme-linked immunosorbent assay; WB: Western blotting; OGD: oxygen-glucose deprivation.

**Figure 2:** Identification of overlapping DEGs. The Venn diagram of DEGs among GSE24519, GSE60993, GSE66360, and GSE97320.The coincident part represents the DEGs shared by the four datasets. Notes: DEGs: differentially expressed genes.

The article "Inflammation and Oxidative Stress Role of S100A12 as a Potential Diagnostic and Therapeutic Biomarker in Acute Myocardial Infarction" was retracted in 2023. Reasons: signs of a paper mill; compromised peer review; unreliable results or conclusions.

**Figure 3:** GO, KEGG, and GSEA analyses of the DEGs and S100A12 in AMI. (a) Biological process (BP). (b) Cellular component (CC). (c) Molecular function (MF). (d) KEGG pathways. (e) GSEA analysis of S100A12. Notes: S100A12: S100 calcium-binding protein A12; AMI: acute myocardial infarction; DEGs: differentially expressed genes; KEGG: Kyoto Encyclopedia of Genes and Genomes; GO: Gene Ontology; GSEA: gene set enrichment analysis.

**Figure 4:** Different expression levels of S100A12 in the AMI group and non-AMI group as well as PPI network of the top 40 DEGs. (a) PPI network, (b) GSE24519, (c) GSE60993, (d) GSE66360, (e) GSE97320, and (f) GSE48060. Notes: PPI node color represents DEGs degree (number of connections), where darker orange indicates more degree. Compared with the non-AMI group, ^∗^*p* < 0.05, ^∗∗^*p* < 0.01, and ^∗∗∗^*p* < 0.001. S100A12: S100 calcium-binding protein A12; PPI: protein-protein interaction; AMI: acute myocardial infarction; DEGs: differentially expressed genes.

**Figure 5:** Comprehensive analysis of S100A12 in AMI. (a) Forest plot of SMD of the included study. (b) Egger's test. (c) SROC curve. Notes: S100A12: S100 calcium-binding protein A12; AMI: acute myocardial infarction; SMD: standardized mean difference; SROC: summary receiver operating characteristics.

**Figure 6:** ROC curve of S100A12 between AMI patients and non-AMI patients based on 5 datasets included, and prediction of miRNAs targeting S100A12. (a) GSE97320, (b) GSE48060, (c) GSE66360, (d) GSE60993, (e) GSE24519, and (f) GSE48060 for AMI prognosis. (g) Venn diagram for miRNA prediction. Notes: S100A12: S100 calcium-binding protein A12; ROC: receiving operator characteristic; AMI: acute myocardial infarction.

**Figure 7:** Establishment of in vitro model of OGD and implementation of S100A12 knockdown/overexpression. (a) CCK-8 assay was used to gauge AC16 cell viability (*n* = 3, per group). (b) The mRNA expression level of S100A12 in Con and OGD groups. (c and d) The protein expression level of S100A12 in Con and OGD groups (*n* = 3, per group). (e) The mRNA expression level of S100A12 in Con, Con+Si-NC, and Con+Si-S001A12 groups (*n* = 3, per group). (f and g) The protein expression level of S100A12 in Con, Con+Si-NC, and Con+Si-S100A12 groups (*n* = 3, per group). (h) The mRNA expression level of S100A12 in Con, Con+OE-NC, and Con+OE-S100A12 groups (*n* = 3, per group). (i and j) The protein expression level of S100A12 in Con, Con+OE-NC, and Con+OE-S100A12 groups (*n* = 3, per group). Notes: S100A12: S100 calcium-binding protein A12; OGD: oxygen-glucose deprivation; Con: control; Si: small interfering; OE: overexpression; SD: standard deviation. Data were presented as mean ± SD based on at least three independent experiments.^∗^*p* < 0.05, ^∗∗^*p* < 0.01, and ^∗∗∗^*p* < 0.001.

The article "Inflammation and Oxidative Stress Role of S100A12 as a Potential Diagnostic and Therapeutic Biomarker in Acute Myocardial Infarction" was retracted in 2023. Reasons: signs of a paper mill; compromised peer review; unreliable results or conclusions.

**Figure 8:** The effect of S100A12 knockdown on inflammation and oxidative stress in OGD model. (a) CCK-8 assay was used to gauge AC16 cell viability in Con+Si-NC, Con+Si-S100A12, OGD+Si-NC, and OGD+Si-S100A12 groups (*n* = 3, per group). (b and c) The protein expression level of S100A12 in the above four groups (*n* = 3, per group). (d) The level of TNF-*α* in the above four groups (*n* = 3, per group). (e) The level of IL-1*β* in the above four groups (*n* = 3, per group). (f) The level of MDA in the above four groups (*n* = 3, per group). (g) The ROS production was detected by the DCFH-DA in the above four groups (*n* = 3, per group) (magnification ×400, scale bar = 200 *μ*m). Data were presented as mean ± SD based on at least three independent experiments. Notes: S100A12: S100 calcium-binding protein A12; OGD: oxygen-glucose deprivation; Con: control; Si: small interfering; SD: standard deviation; DCFH-DA: dichlorodihydrofluorescein diacetate. ^∗^*p* < 0.05, ^∗∗^*p* < 0.01, and ^∗∗∗^*p* < 0.001.

**Figure 9:** The effect of S100A12 overexpression on inflammation and oxidative stress in OGD model. (a) CCK-8 assay was used to gauge AC16 cell viability in Con+OE-NC, Con+Si-S100A12, OGD+OE-NC, and OGD+OE-S100A12 groups (*n* = 3, per group). (b and c) The protein expression level of S100A12 in the above four groups (*n* = 3, per group). (d) The level of TNF-*α* in the above four groups (*n* = 3, per group). (e) The level of IL-1*β* in the above four groups (*n* = 3, per group). (f) The level of MDA in the above four groups (*n* = 3, per group). (g) The ROS production was detected by the DCFH-DA in the above four groups (*n* = 3, per group) (magnification ×400, scale bar = 200 *μ*m). Data were presented as mean ± SD based on at least three independent experiments. Notes: S100A12: S100 calcium-binding protein A12; OGD: oxygen-glucose deprivation; Con: control; Si: small interfering; SD: standard deviation; DCFH-DA: dichlorodihydrofluorescein diacetate. ^∗^*p* < 0.05, ^∗∗^*p* < 0.01, and ^∗∗∗^*p* < 0.001.

**Table 1:** The datasets of AMI in GEO database.

Accession	Author	Year	Country	Platform	Non-AMI	AMI
GEO: GSE24519	Bellin M	2017	Italy	GPL2895	4	34
GEO: GSE48060	Suresh R	2014	USA	GPL570	21	31
GEO: GSE60993	Eun JW	2015	South Korea	GPL6884	7	17
GEO: GSE66360	Kramer ER	2015	USA	GPL570	50	49
GEO: GSE97320	Meng F	2017	China	GPL570	3	3

Notes: AMI: acute myocardial infarction; GEO: Gene Expression Omnibus.

The article "Inflammation and Oxidative Stress Role of S100A12 as a Potential Diagnostic and Therapeutic Biomarker in Acute Myocardial Infarction" was retracted in 2023. Reasons: signs of a paper mill; compromised peer review; unreliable results or conclusions.

**Table 2:** The significant gene ontology and signal enrichment terms of S100A12 in biological process category.

Term	Count	Genes	*p* value
GO:0006954~inflammatory response	17	SYK, IL37, GPR68, TNFRSF18, LY96, TNFRSF10B, CYBA, PTGS2, TIRAP, MMP25, NFKBIZ, S100A12, CCL2, TLR8, CD14, LTBR, and KLRG1	0.013
GO:0043123~positive regulation of I-kappaB kinase/NF-kappaB signaling	9	UBE2I, PELI2, MIER1, PELI1, S100A12, TNFRSF10B, LTBR, TIRAP, and LTF	0.031
GO:0043406~positive regulation of MAP kinase activity	5	EDN1, LRRK2, S100A12, PSEN1, and VEGFA	0.045

**Table 3:** Characteristics of the datasets included in the study.

Author (publication year)	Country	Data source	Platform	Non-AMI			AMI		
				N0	M0	SD0	N1	M1	SD1
Bellin M (2017)	Italy	GEO: GSE24519	GPL2895	4	1.020	0.104	34	2.758	2.003
Suresh R (2014)	USA	GEO: GSE48060	GPL570	21	11.025	0.672	31	11.826	0.871
Eun JW (2015)	South Korea	GEO: GSE60993	GPL6884	7	9.728	0.459	17	11.163	1.087
Kramer ER (2015)	USA	GEO: GSE66360	GPL570	50	6.404	1.414	49	9.386	1.984
Meng F (2017)	China	GEO: GSE97320	GPL570	3	3.166	0.102	3	10.224	0.567

Notes: AMI: acute myocardial infarction; N: number; M: mean; SD: standard deviation.

## Data Availability

The datasets supporting the conclusions of this study are included in the article.

## Abbreviations

AMI: Acute myocardial infarction
S100A12: S100 calcium-binding protein A12
GEO: Gene Expression Omnibus
KEGG: Kyoto Encyclopedia of Genes and Genomes
GO: Gene Ontology
SMD: Standardized mean difference
ROC: Receiver operating characteristic
SROC: Summary receiver operating characteristic
GSEA: Gene set enrichment analysis
RT-qPCR: Real-time quantitative PCR
ELISA: Enzyme-linked immunosorbent assay
WB: Western blotting
OGD: Oxygen-glucose deprivation.

## Supplementary Materials

Supplementary Materials Supplementary Table 1: the S100A12-specific sequence of knockdown and overexpression in this study.
